This article has been retracted.

# The Role of Cavin3 in the Progression of Lung Cancer and Its Mechanism

**DOI:** 10.1155/2020/6364801

**Published:** 2020-04-14

**Authors:** Gaozhong Sun, Kewei Ni

**Affiliations:** Department of Cardio-Thoracic Surgery, Zhejiang Provincial People's Hospital, People's Hospital of Hangzhou Medical College, 158 Shangtang Road, Hangzhou, 310014 Zhejiang, China

## Abstract

**Objective:**

The purpose of this study was to describe the role of Cavin3 in the progression of lung cancer and its underlying mechanism.

**Methods:**

Totally, 200 cases of lung cancer tissues and corresponding paracancer tissues were collected. Cavin3 expression in samples was determined by qRT-PCR, and the correlation with lung cancer stages as well as prognosis was statistically analyzed combined with matched clinical information. To investigate the mechanism of Cavin3 in lung cancer progression, firstly, Cavin3 was detected in lung cancer cell lines A549, PC9, and H520. Then, cells with stable Cavin3 overexpression and Cavin3 knockout were established to determine the effect of Cavin3 overexpression on the mammalian target of rapamycin (mTOR) signaling pathway. Subsequently, cells were harvested for cell proliferation, migration, and invasion assays *in vitro*, as well as nude mouse transplantation tumor experiment *in vivo*.

**Results:**

Cavin3 was seen to be highly expressed in cancer tissues. Statistical analysis with matched clinical data showed that Cavin3 as a prognostic indicator of lung cancer had important clinical value. In addition, it could be found that high expression of Cavin3 was able to promote cell proliferation, migration, and invasion and also potentiate tumor formation *in vivo*.

**Conclusion:**

Cavin3 was highly expressed in lung cancer, and it was capable to promote cell proliferation, invasion, and migration.

## 1. Introduction

Lung cancer is one of the most serious malignancies threatening people's health and life, and it has become a public health issue of great concern throughout the world [1]. In 2018, lung cancer accounts for 11.6% of the total cancers globally, and it is the leading cause for cancer death with 18.4% of the total [2]. In the past decades, with the deepening of research on new therapeutic targets for lung cancer, individualized clinical treatment has been widely applied [3]. However, the survival rate remains poor of only about 15% [4]. Therefore, for better efficacy and prognosis, it is crucial to clarify the molecular mechanism as well as explore effective biomarkers in lung cancer tumorigenesis and development.

A variety of cellular signaling pathways were shown to be involved in the lung cancer progression, among which the mammalian target of rapamycin (mTOR) signal also exhibits a vital role in many other tumors as proved by a large amount of evidence [5]. The mTOR pathway composed of multiple feedback loops can be used as a promising target in cancer treatment, but the underlying mechanism is not clear. In our previous study on signal molecule DEPTOR (endogenous mTOR inhibitor) in lung cancer, we found that Cavin3 was an important protein involved in the mTOR signaling pathway. Thus, we speculated that Cavin3 may play an important role in lung cancer progression. However, the effect of Cavin3 on tumorigenesis and development has not been further studied, which enables us to make more efforts on the underlying mechanism and to clarify the relationship between Cavin3 and mTOR signaling pathway.

The present study intended to verify the overexpression of Cavin3 in numerous samples of lung cancer based on the previous studies, then investigate the role of Cavin3 in tumorigenesis and development to excavate the underlying mechanism, thereafter evaluate the possibility of Cavin3 serving as a prognostic indicator or a promising therapeutic target. Our study would help us know more about Cavin3 in cancer progression, providing a new avenue for the targeted therapy in lung cancer.

## 2. Materials and Methods

### 2.1. Materials

Human lung cancer cell lines A549 and H520 were purchased from the Cell Resource Center of Institute of Basic Medical Sciences, Chinese Academy of Medical Sciences, with resource numbers 3111C0001CCC000002 and 3111C0001CCC000197, respectively. PC9 (No. CM-H210) was from Gaining Biology. PrimeScript RT Kit (No. RR047a) was from TaKaRa. qPCR Kit (No. RT-02111) was from Shanghai FanKe Biotechnology Co., Ltd. RPMI-1640 medium was from Sigma. Primary antibodies and horseradish peroxidase- (HRP-) labeled secondary antibody used in Western blot were from Abcam, UK. Lipofectamine™ 2000 and TRIzol lysate were from Invitrogen. The BCA quantitative kit was from Multi Sciences (Lianke) Biotech, Co., Ltd. Transwell inserts were from Millipore, USA, and the protein immunoprecipitation kit was from Pierce, USA. The eukaryotic expression vector and Cavin3-mRFP as well as Cavin3-shRNA knocked out by Cavin3 were produced by Addgene, USA.

### 2.2. Methods

#### 2.2.1. Clinical Data

200 cases of lung cancer tissues and corresponding paracancer tissues were collected at Zhejiang Provincial People's Hospital from January 2014 to September 2016. Informed consent was written informed consent. All patients had not been treated with preoperative radiotherapy or chemotherapy. Cancer samples were taken from the intraoperative tumors, and adjacent cases were from the normal tissues 5 cm away from the tumor [6]. All cancer tissues composed of greater than 70% cancer cells and were histopathologically diagnosed. Samples extracted were immediately put into RNA preservation solution, with a part paraffin-embedded as well as sliced (4 *μ*m) and the other part stored under -80°C. In this study, except those who died of other diseases or accidents, the clinical and previous follow-up data of all other patients were well documented and available. Thus, these patients were scheduled a follow-up for 60 months and analyzed in survival using the Kaplan-Meier method. The period beginning at treatment and ending at death is defined as the overall survival (OS). During the follow-up, tumor relapse or patients' death was the end point; otherwise, the final follow-up time was defined as the end. This project had got the informed consent of all subjects, and the acquisition as well as the use of tissue samples was approved by the Ethics Committee in Zhejiang Provincial People's Hospital.

#### 2.2.2. Real-Time Quantitative PCR (qRT-PCR)

TRIzol was used to extract total RNAs from cancer tissues and paracancer tissues. An ultraviolet spectrophotometer was applied to determine the RNA concentration. PrimeScript RT Kit was employed for the cDNA synthesis through reverse transcription. All primers were designed using Primer 5.0 software: Cavin3: forward primer: 5′-CACGTTCTGCTTCAAGGAG-3′, reverse primer: 5′-TGTACCTTCTGCAATCCGGTG-3′; *β*-actin: forward primer: 5′-ATCCGTAAGGACCTGTATGCCAAC-3′, reverse primer: 5′-GATCCATGTTGTTGAAGGGTGGA-3′.

qRT-PCR was carried out following the instructions of the qPCR kit. The reaction conditions were as follows: predenaturation at 95°C for 5 min, 30 cycles of 95°C for 40 s, 57°C for 40 s, and 72°C for 40 s, followed by extension at 72°C for 10 min and 4°C for 5 min. 2^-*ΔΔ*Ct^ was used to express the relative transcriptional level of the target mRNA, therein ΔCt = Ct (target gene)–Ct (internal reference gene). Each experiment was repeated three times, and the results were averaged.

#### 2.2.3. Cell Culture and Transfection

A549 cells were cultured in RPMI-1640 medium containing 10% fetal bovine serum (FBS) with 5% CO_2_ at 37°C. Cells in the logarithmic phase were seeded into 6-well plates at a density of 5 × 10^5^ cells/well one day before transfection and divided into four groups: blank group, Cavin3-mRFP group, Cavin3-shRNA group, and Cavin3-shNC group. A549 cells with stable Cavin3 overexpression or low expression were constructed using lentivirus vectors. After being extracted and sequenced, the eukaryotic expression vector of Cavin3 and its shRNA was constructed. Three packaging plasmids (Cavin3-mRFP, Cavin3-shRNA, and Cavin3-shNC) were cotransfected with the expression vector into A549 using Lipofectamine 2000 (Invitrogen, USA). All cells were maintained in 5% CO_2_ at 37°C. After 6 h, cells were grown for another 48 h in fresh mediums. The sequence of Cavin3-shRNA: sense sequence: 5′-CACCG GTTGA AAGGG CATTC CGTGA CTCGA GTCAC GGAAT GCCCT TTCAA CC-3′; antisense sequence: 5′-AAAAG GTTGA AAGGG CATTC CGTGA CTCGA GTCAC GGAAT GCCCT TTCAA CC-3′ and Cavin3-shNC: sense sequence: 5′-TGCTT CATAA GGCGC ATAGC TTCAA GAGAG CTATG CGCCT TATGA AGCTT TTTTC-3′; antisense sequence: 5′-TCGAG AAAAA AGCTT CATAA GGCGC ATAGC TCTCT TGAAG CTATG CGCC T TATGA AGCA-3′.

#### 2.2.4. CCK-8

Transfected cells were digested with trypsin and prepared to the cell suspension with a concentration of 1.5 × 10^4^ cells/ml. Then, the cells were planted at 3 × 10^3^ cells/well into 96-well plates in 5% CO_2_ at 37°C. Ten reduplicative plates were set for the avoidance of contingency. When cells' attachment occurred, cells at 24, 48, 72, and 96 h were incubated with 10 *μ*l of CCK-8 solution for another 4 h, respectively. The absorbance value of each well was read at 450 nm in wavelength on the enzyme-labeled instrument. The cell growth curve was plotted, with time as abscissa and absorbance value as ordinate. (The OD values of all times are the results of subtracting the initial OD values.)

#### 2.2.5. Transwell Migration and Invasion Assay

Transwell inserts (8 *μ*m, dedicated for 24-well plates) were used to detect cell migration and invasion ability. Inserts used in the invasion assay were precoated with a layer of artificial Matrigel Matrix (prepared by ECM gel and serum-free RPMI-1640 medium; 1 : 19) in the upper chamber. Cells were cultured in serum-free RPMI-1640 medium and prepared to cell suspension (2 × 10^5^ cells/ml in invasion assay and 10^5^ cells/ml in migration assay). Thereafter, 200 *μ*l of cell suspension was added to the upper chamber, and the RPMI-1640 medium containing 9% FBS with a total volume of 600 *μ*l was added to the lower chamber. All cells were maintained in 5% CO_2_ at 37°C. After 24 hours, cells migrated or invaded were fixed by polyformaldehyde and stained using crystal violet. Images were captured under a microscope, and the cells in each field were counted. Four regions were selected to calculate the number of cells successfully invading the lower chamber.

#### 2.2.6. Western Blot

Cells were washed in PBS before experiment. 0.1 ml-1 ml of total protein extraction reagent (or nucleoprotein extraction reagent) containing protease inhibitor was utilized to isolate total proteins (or nucleoproteins) from the cells, and the BCA protein quantitation kit was applied to determine the protein concentration. Subsequently, the protein samples were separated by SDS-PAGE together with the prestained protein marker and then transferred onto the PVDF membrane overnight at 30 mA at 4°C, following the instructions of Bio-Rad Trans-Blot Turbo Transfer System. After being blocked in 5% skim milk at room temperature for 1 h, the membrane was incubated with primary antibodies at room temperature for 1.5 h, followed by horseradish peroxidase- (HRP-) labeled secondary antibody at room temperature for 1 h. GAPDH was taken as the internal control. Protein bands were detected by chemiluminescence and exposed as well as visualized on X-ray films. GIS1000 analysis software was employed to digitalize the grey scan values of the protein bands.

#### 2.2.7. Nude Mouse Transplantation Tumor Experiment

Cavin3-shNC and Cavin3-shRNA were stably transfected into A549 cells, respectively. Then, the transfected cells were planted under the armpit of nude mice, and the tumor growth status was observed weekly. When the tumors were grown to be visible to the naked eyes, a vernier caliper was utilized to measure the long and short diameters. Tumor weight was calculated according to the following formula: tumor weight (*μ*g) = long diameter (mm) × short diameter (mm)^2^/2, and the tumor growth curve was plotted accordingly. Four weeks later, the nude mice were executed and images of tumors in each group were captured for further comparison. All procedures conformed to the convention released by the International Council for Laboratory Animal Science and meet the correlated national standard.

#### 2.2.8. Statistical Analysis

All the data were processed by SPSS 21.0 statistical software. The measurement data were presented as the form of mean value ± standard deviation. The comparison between two groups was analyzed by *t*-test, and the comparison among multiple groups was analyzed by one-way analysis of variance (ANOVA). The count data were expressed as a percentage or rate and compared using the *χ*^2^ test. Comparison among multiple count data was performed using ANOVA and validated by homogeneity testing of variance. Data at different time points were compared using repeated-measures ANOVA. The Kaplan-Meier method was applied to analyze the survival of patients. *p* < 0.05 was considered statistically significant.

## 3. Results

### 3.1. Expression of Cavin3 in Lung Cancer Tissues [7]

qRT-PCR was conducted to investigate the alteration of Cavin3 in lung cancer tissues. As shown in Figure 1, Cavin3 in lung cancer tissues was significantly upregulated relative to that in paracancer tissues (*p* < 0.05).

### 3.2. Relationship between Cavin3 and Clinical Pathological Parameters of Lung Cancer

In order to clarify the role of Cavin3 in clinical diagnosis of lung cancer, the relationship between Cavin3 and clinical pathological parameters was investigated. The median value of Cavin3 expression was set as the threshold for the high and low expression classifications. As revealed in Table 1, high expression of Cavin3 was observed to be associated with TNM staging, tumor size, and lymph node metastasis, with a statistically significant difference (*p* < 0.05). However, no correlation with age, gender, smoking history, and histological classification was suggested, and the difference was with no statistical significance (all *p* > 0.05). These results indicate that the expression level of Cavin3 is closely related to tumor progression, and it is also a risk factor for lung cancer.

### 3.3. Relationship between Cavin3 and Lung Cancer Prognosis

Kaplan-Meier analysis was performed to explore the relationship between Cavin3 and prognosis of patients with lung cancer. As indicated in the survival curves plotted in Figure 2, Cavin3 of high expression significantly decreased the overall survival rate in comparison with that of low expression, and the difference was statistically significant (*p* < 0.05).

### 3.4. Relationship between Cavin3 and Lung Cancer Malignant Degrees [8]

Lung cancer cells A549, PC9, and H520 with different biological characteristics were used to further discuss the correlation between Cavin3 and malignant degrees of lung cancer. Western blot revealed that the expression of Cavin3 in lung squamous carcinoma cell line H520 was the lowest, followed by EGFR-TKI-sensitive lung adenocarcinoma (LUAD) cell line PC9, whereas that in undifferentiated LUAD cell line A549 was the highest (Figure 3). In addition, compared with H520, the difference of the Cavin3 expression level was statistically significant (*p* < 0.05). The results showed that the highest expression level of Cavin3 was found in undifferentiated cell lines.

### 3.5. Effect of Cavin3 Expression on the mTOR Signaling Pathway in Lung Cancer Cells

Cells were divided into blank group, Cavin3-mRFP group, and Cavin3-shRNA group. As demonstrated by Western blot shown in Figure 4, compared with the blank group, the p-mTOR protein level in the Cavin3-mRFP group was significantly upregulated (*p* < 0.05), while that in the Cavin3-shRNA group was greatly downregulated (*p* < 0.05). Besides, there was no significant difference in mTOR between the Cavin3-mRFP group and the Cavin3-shRNA group (*p* > 0.05). This result indicates that Cavin3 activates the mTOR signaling pathway.

### 3.6. Effect of Cavin3 Expression on Cell Proliferation

CCK-8 was performed to determine cell proliferation. As plotted in Figure 5, cell proliferation was significantly increased in the Cavin3-mRFP group relative to that in the blank group (*p* < 0.05), whereas that was remarkably decreased in the Cavin3-shRNA group (*p* < 0.05).

### 3.7. Effect of Cavin3 Expression on Cell Invasion and Migration

Transwell was carried out for the assessment of cell invasion and migration. As shown in Figure 6, cells in the Cavin3-mRFP group had greatly increased migration and invasion ability relative to the blank group (*p* < 0.05), whereas in the Cavin3-shRNA group, those were both markedly inhibited (*p* < 0.05).

### 3.8. Effect of Cavin3 Expression on the Tumor Formation of Lung Cancer *In Vivo*

To further validate the promotion of high Cavin3 on lung cancer tumor formation *in vivo*, Cavin3-shNC- and Cavin3-shRNA-transfected A549 cells were planted into nude mice to test the tumor size and weight. Results plotted in Figure 7 showed that compared with the Cavin3-shNC group, the volume and weight of tumors in the Cavin3-shRNA group were both decreased significantly (both *p* < 0.05).

## 4. Discussion

In recent years, lung cancer has showed increased prevalence, usually accompanied by lymph node metastasis, as well as low sensitivity to radiotherapy or chemotherapy and poor prognosis [9]. Studies have reported that the protein level and functional role of Cavin in cancer cells are closely related to cancer metabolism and stress signaling [10, 11]. Moreover, Cavin3 can interact with PP1-*α* and the product functions on cell apoptosis [12], suggesting that Cavin3 may have important research significance on tumorigenesis and development. Also, it has been reported that ROR1-Cavin3 interaction is a necessity for caveola-dependent endocytosis and prosurvival signaling on the cell surface in LUAD [13]. In addition, the aberrant expression of Cavin3 (also known as PRKCDBP) in cancer cells is considered to be a new therapeutic target for non-small-cell lung cancer as revealed by another study [14]. Previously, Cavin3 had been found to be overexpressed in lung cancer, but the role of Cavin3 in lung cancer progression was not particularly clear. Besides, Cavin3 is a part of the mTOR pathway, thus clarifying the effect of Cavin3 on lung cancer occurrence and development which might make it possible for the mTORC1 pathway to be a novel regulatory target in lung cancer [15–17].

In this study, the expression levels of Cavin3 in postoperative cancer samples and matched paracancer tissues were detected, finding the relatively high expression in cancer cases. Further studies had found that Cavin3 was firmly associated with a diversity of malignant biological behaviors in lung cancer, including TNM staging, tumor size, and lymph node metastasis. Kaplan-Meier analysis revealed that high expression of Cavin3 resulted in a significant reduction in overall survival, which was consistent with the finding suggested by Yamaguchi et al. [13]. Furthermore, expression levels of Cavin3 were examined in A549, PC9, and H520 lung cancer cell lines with different biological characteristics. It was found that Cavin3 exhibited the lowest expression in lung squamous cell carcinoma cell line H520, then in EGFR-TKI-sensitive LUAD cell line PC9, and the highest expression in undifferentiated LUAD cell line A549. Thus, it could be concluded that Cavin3 may be positively correlated with the malignant degrees of lung cancer cells. In addition, tests on biological behaviors of lung cancer cells were conducted after upregulating/downregulating Cavin3 expression and demonstrated that high expression of Cavin3 promoted cell proliferation, invasion, and metastasis, further validating its regulatory role in lung cancer. Furthermore, Cavin3 was also proved to be able to potentiate tumor formation in lung cancer *in vivo*.

This study described the important role of Cavin3 in lung cancer clinical diagnosis and in the proliferation, invasion, and metastasis of cancer cells. However, the underlying mechanism is worthy of further research. Also, more efforts should be put in exploring the potential target of Cavin3 in the mTOR signaling pathway in lung cancer.

In conclusion, Cavin3 is involved in the tumorigenesis, development, cell invasion, and metastasis in lung cancer. It can be used as one of the clinical indicators to evaluate the malignant biological behaviors of lung cancer, which helps to find the potential target of Cavin3 in the mTOR signaling pathway in lung cancer.

## Figures and Tables

**Figure 1:** Differential expression of Cavin3 in lung cancer tissues and paracancer tissues. Note: *N* = 200, ∗ means *p* < 0.05.

**Figure 2:** Survival analysis of Cavin3 in lung cancer.

**Figure 3:** Differential expression of Cavin3 in lung cancer cell lines with different biological characteristics. (a) Protein bands of Cavin3 in different lung cancer cells lines and (b) corresponding expression levels (∗ means *p* < 0.05).

**Figure 4:** Effect of Cavin3 expression on the mTOR signaling pathway in lung cancer cells. (a) Protein bands of mTOR pathway-related proteins and (b) corresponding expression levels (∗ means *p* < 0.05, *N* = 200).

**Figure 5:** Cell growth curve in lung cancer. Note: ∗ means *p* < 0.05, *N* = 3.

**Figure 6:** Effects of Cavin3 expression on the cell invasion and migration in lung cancer. Images of (a) cell migration and (b) invasion in each transfected group and (c: migration, d: invasion) corresponding histograms (∗ means *p* < 0.05, *N* = 3).

**Figure 7:** Tumor formation of lung cancer in nude mice *in vivo*. (a) Pictures of transplanted tumors and corresponding (b) growth curves of tumor volume as well as (c) histogram of tumor weight (∗ means *p* < 0.05, *N* = 2).

**Table 1:** Relationship between the expression of Cavin3 and clinicopathological characteristics of lung cancer.

Group	*N* = 200	Relative expression level of Cavin3		*p*
		High expression	Low expression	
Age
<60	101	56	45	0.12
≥60	99	44	55	
Gender				
Male	108	52	56	0.57
Female	92	48	44	
Size				
<3 cm	105	45	60	0.034
≥3 cm	95	55	40	
Lymph node metastasis				
None	96	41	55	0.048
Exist	104	59	45	
Smoking history				
None	80	43	37	0.39
Exist	120	57	63	
TMN stage				
I-II	97	41	56	0.034
III-IV	103	59	44	
Histological classification				
Lung adenocarcinoma	112	55	57	0.78
Lung squamous carcinoma	88	45	43	

## Data Availability

The data used to support the findings of this study are available from the corresponding author upon request.
